# Ameliorative effects of crocin on paraquat-induced oxidative stress in testis of adult mice: An experimental study

**DOI:** 10.18502/ijrm.v17i10.5490

**Published:** 2019-11-28

**Authors:** Fahime Sadat Kamali, Rasoul Shahrooz, Golamreza Najafi, Mazdak Razi

**Affiliations:** ^1^Department of Histology and Embryology, Faculty of Veterinary Medicine, Urmia University, Urmia, Iran.; ^2^Department of Anatomy and Embryology, Faculty of Veterinary Medicine, Urmia University, Urmia, Iran.

**Keywords:** Histology, Testis, Paraquat, Crocin, Mice.

## Abstract

**Background:**

Paraquat (PQ), as a pyridine compound, is widely used worldwide to control annual weeds. The oxidative stress caused by PQ can cause deleterious changes in the testicular tissue.

**Objective:**

An investigation on the protective effects of Crocin (CCN) against PQ-induced oxidative damages and apoptotic indices in testicular tissue.

**Materials and Methods:**

Twenty-eight adult male albino mice (20-25 gr) were divided into four groups (n = 7/each). The control group received 0.1 ml/day of normal saline by intraperitoneal injection (IP); sham-control group received PQ 5 mg/kg/day, IP, and the experimental groups received PQ (CCN+PQ) and CCN-sole (200 mg/kg/day, IP), respectively, for 35 continuous days. At the end of the treatment period, the testes were dissected out and used for biochemical, molecular, and histological analyses. The expressions of tumor suppressor *p53*, B-cell lymphoma 2 (*bcl-2*), and *caspase-3* were considered as hallmark factors of mitochondria-dependent apoptosis. Moreover, the testicular superoxide dismutase (SOD) and malondialdehyde (MDA) were evaluated as key biomarkers for oxidative stress.

**Results:**

The PQ significantly (p < 0.02, p < 0.01) diminished the spermatogenesis indices and SOD, increased MDA levels, and enhanced the apoptosis-related gene expression. However, the co-administration of CCN and PQ significantly (p < 0.01, p < 0.01, p < 0.02) ameliorated the spermatogenesis ratio, upregulated the SOD level as well as *bcl-2* expression, and reduced the MDA content and apoptosis vs the PQ-sole group.

**Conclusion:**

This study showed that the antioxidant properties of CCN enable to ameliorate the PQ-induced destructive effects by upregulating the testicular structure, antioxidant and apoptotic status.

## 1. Introduction 

Paraquat (PQ) as a safe herbicide is widely used in agriculture, however a dermal contact or spray exposure can generally cause limited and localized injury (1), and a casual or deliberate ingestion has an extremely high mortality rate (2). For this reason, PQ has been restricted in some countries. It is available in rural areas of countries then and is a common case for intentional self-poisoning (3). The PQ, N, N'-dimethyl-4,4'-bipyridinium dichloride, an organic agent with the chemical formula of [(C6H7N)2]Cl2, is one of the most common agricultural herbicides. The PQ is known as one of the main biorisk-factors in the ecosystem in addition to its role of being a pesticide (4). The alveolar cells of the lung selectively absorbs PQ (*5*). The PQ results in lung fibrosis and has been reported to lead death by asphyxiation (6). In another study, the PQ has shown to result in Parkinson's disease in farm workers (7). In line, the PQ toxicity in rats has been known as a model to induce Parkinson's-like neurological degenerative disease (8). Moreover, the chronic exposure to PQ has been reported to result in severe oxidative stress by interacting in REDOX system (9). In line with this issue, it is well established that the junction between endothelial cells as well as, germ cell DNA integrity in testicles are sensetive against high amount of free radicals (10). After the testis torsion/detorsion, the level of peroxidative damage observed in testicular tissue cause a biochemical reperfusion injury (11, 12). A study showed that the pretreatment with antioxidants may be ameliorate the oxidative stress induced by testicular torsion/detorsion (11). It has been also showed that the administration of vitamin C within 5hr after the testicular torsion improved the histological parameters and testosterone levels (13). Furthermore, another study showed that the testis histomorphometrical parameters significantly ameliorated in the testicular torsion after receiving an extract of *Syzygium aromaticum* in comparison to the torsion/detorsion (TD) group (14). Stress oxidative induced by the experimental debate that disturbed the Johnson core, the diameter of seminiferous tubules and sperm parameters in rat's testis, is alleviated by the administration of *G. officinalis *extract (15).

In line with male infertility disorders, it has been shown that PQ adversely affects the spermatogenesis (16), reduces the sperm quality, including count, motility, and morphology (4), and results in chromosomal aberrations in spermatozoa, spermatid, and preleptotene spermatogonial cells (17). Spermatogenesis is a dynamic system, which is characterized by cell proliferation and differentiation. Similar to hypermitotic tissues, the physiologic cellular proliferation of testicular tissue is maintained with controlled apoptosis. Indeed, the apoptosis is processed through intrinsic (mitochondria-dependent) and extrinsic (death receptor Fas and Fas-ligand-dependent) pathways (18).

Crocin (CCN) has attracted scientific attention and finally found a considerable place in pharmaceutical science due to its anti-inflammatory, antioxidant (19), anti-spasm (20), anti-depression (21), anti-cancer (22) and neuroprotective properties (23). A study showed that the CCN increases antioxidant enzymes and testosterone. However, it reduced testicular histological destructive changes in CP-treated mice (24).

Considering the oxidative stress as the main mechanism of PQ action and minding the adverse effect of free radicals on mitochondrial membrane integrity, the current study was performed to investigate the protective effect of CCN against PQ-related derangements.

## 2. Materials and Methods

### Chemicals

The PQ, with the formulation of SL20%, was taken from EXIR Co. (Tehran, Iran) and the CCN was obtained from Sigma-Aldrich Co. (Cas NO: 17304, St. Louis, MO, USA). Commercial kits for superoxide dismutase (SOD) was obtained from RANDOX reagents Co. (Rondaxlab, Crumlin, BT 29, UK). All other chemicals were commercial products of analytical grade.

### Animals and grouping

To perform the current original study, 28 mature Albino mice (20-25 gr) were randomly divided into 4 control and experimental groups (n = 7/each). The animals received food and water at libitum, in a standard light/dark and temperature condition.

1) The control group (Con) received 0.1 ml/day, IP of normal saline. 2) CCN-sole group received only CCN (200 mg/kg /day, IP) (25). 3) The sham-control group (PQ), received PQ (5 mg/kg/day, IP) (26). 4) The experimental group (PQ+CCN), received CCN (200 mg/kg/day, IP) along with PQ. All four groups were treated for 35 continuous days.

### Tissue sampling and weight determination

Following the test termination, the animals were euthanized by overdose administration of ketamine and xylazine (Alfasan, Woerden, the Netherland) (three times more than the anesthesia dose of ketamine 120 mg/kg and xylazine 15 mg/kg). The total body weights of animals were recorded before and after the trial. Moreover, after the trial, the testicular weights as well as testicular weight relative to the total body weight were determined and compared between the groups. Next, the left testes were considered for further molecular and biochemical analyses at -70°C. The right testicles were fixed in 10% formal saline for further histological and morphometric studies.

### Histological analyses

Following fixation (72 hr), routine tissue passage and paraffin embedding were conducted. Then, the samples were cut (5-6 µm) using a rotary microtome (Lites, Germany). The histomorphometric analyses were performed after Hematoxylin-Eosin staining. For this purpose, the tubular repopulation (RI), differentiation (TDI) and spermiogenesis (SPI) indices were analyzed. The seminiferous tubules with more than 3 layers were marked as those tubules with positive TDI. Moreover, the those seminiferous tubules with developing spermatozoa were marked as tubules with positive SPI. Moreover, the seminiferous tubules with high percentages of active spermatogonia (with a dark nucleus) were considered as positive RI. Finally, the percentages of tubules with positive TDI, SPI, and RI were evaluated in 3 cross sections from each animal (total 21 cross sections from each group). Moreover, the Leydig and Sertoli cell distribution *per* mm${}^{2}$ of testicular tissue were counted in 3 cross sections from each animal (total 21 cross sections from each group).

The histological photomicrographs were taken using an onboard camera (SONY Zeiss, Cyber-Shot, Japan) and edited/combined with Adobe Photoshop CS10 (Adobe System Inc., Mountain View, CA, USA).

### Assessment of testicular antioxidant status

In order to evaluate the biochemical activity of the SOD and malondialdehyde (MDA) content in testicular tissue, the tissue samples were weighed and 0.6 gr of each tissue were homogenized in 10 volumes of ice-cold 50 mM potassium phosphate buffer (pH 7.4) with 0.3 M KBr and a set of antiproteolytic agents (containing: 0.5 mM phenyl methylsulfonyl fluoride, 3 mM diethylenetriaminepentaacetic acid, 90 mg of aprotinin l${}^{-1}$, 10 mg of pepstatin l${}^{-1}$, 10 mg of chymostatin l${}^{-1}$, and 10 mg of leupeptin l${}^{-1}$). Thereafter, the SOD activity of homogenates was assayed by using commercial standard kits (ZB-SOD-96A, Zellbio, GmbH). Finally, the rates of absorbance for samples were measured at 420 nm and compared between the groups. The MDA contents of testicles were measured by using the thiobarbituric acid (TBA) reaction as described previously and the absorbance rates of samples were measured at 532 nm (27). Finally, the MDA was evaluated based on the Lowry technique (28) and the results for MDA was presented based on nmol/mg of tissue.

### RNA isolation and semi-quantitative reverse transcriptase polymerase chain reaction (RT-PCR)

To perform RT-PCR test, 0.3 gr from each sample (n = 7 from each group) were used for RNA extraction by using TRIzolⓇ-based total RNA isolation kit (GIBCO BRL, Gaithersburg, Maryland, USA). Next, the quality and concentration of extracted mRNA were evaluated by NanoDrop-1000 spectrophotometer (Thermo Scientific, Washington, USA) at 260 nm and A260/280 = 1.8-2.0 and stored in -70${}^{\circ }$C. “The cDNA was prepared by using 1 µg of RNA from each sample and used as a template for the amplification by the PCR with the specific forward and reverse primers presented in Table I. The PCR amplification conditions were 35-40 cycles of 95°C for 20 sec; annealing temperature [50°C for *caspase-3* (45 s), 62°C for *Bcl-2* (1 min), 59°C for Bax (1 min), 52°C for *p53* (1 min), and 57°C for GAPDH (1 min)]; elongation: 72°C for 1 min and 72°C for 5 min. Speciﬁc primers (29) were designed and manufactured by Gen-Fanavarn Co. (Tehran, Iran). The amplified products (10 µl, including 7 µl from the sample and 3 µl from loading buffer) were electrophoresed in 1.5% agarose gels, stained with ethidium bromide, and viewed using ultraviolet (UV) trans-illuminator (ATP technology, Iran) and visualized by Gel-Pro analyses software (ATP, version 2.1 for window 7). In order to quantify the target gene amplification, the ratio between product genes and the GAPDH (internal control) was calculated to normalize (30).

### The DNA ladder test

To assess DNA fragmentation the DNA ladder was performed using Cina Pure-DNA extraction kit (Sinaclon, Iran). In this process, 35 mg of testicles was homogenized with 100μl protease buffer in the microcentrifuge tubes. Then, incubation of the tubes at 55°C for 2hr has been down. Next, 100 μl of samples were added into the new microtubes and precipitated with 300μl of precipitation solutions (isopropanol based) for 5min and centrifuged (12000 g) for 10 min. The tubes were decanted and placed on a tissue paper for 2-3 sec and 1 ml buffer solution (ethanol-based) was added to pellets and mixed through 5-sec. following centrifugation (2xafter the supernatant was poured off and the pellets were dried at 65°C for 5 min. Finally, the unsolved residues were precipitated by centrifugation at 12,000 g for 30 sec and the DNA containing supernatant was removed. The DNA content was assessed using a NanoDrop-1000 spectrophotometer (Thermo Scientific, Washington, USA). Then, the DNA quantity was estimated and a volume of 2μg DNA (15-17μl of eluted DNA) was added to the loading buffer (50% glycerol, 2 mm ethylenediaminetetraacetic acid, and 0.40% bromophenol blue), and DNA solution was loaded on a 1% agarose gel (70-V constant voltage, 70 min). The PST1 was used as a marker to identify the DNA amount. Gels were stained with ethidium bromide and visualized by Gel Doc 2000 system (ATP, Tehran, Iran).

**Table 1:** Nucleotide sequences, product size for primers used in RT-PCR


**Target gene**	**Primer sequences (5'-3')**	**Product size (bp)**
*bcl-2*	Forward: GCGAAGTGCTATTGGTACCTG Reverse: ATATTTGTTTGGGGCAGGTCT	350
*p53*	Forward: CTCTCCTCCCCTCAATAAGC Reverse: AAACACGAACCTCAAAGCTG	650
*caspase-3*	Forward: TGACTGGAA AGCCGA AACTC Reverse: AGCCTCCACCGGTATCTTCTV	610
GAPDH	Forward: CTTCCTCCTCAGACCGCTTT Reverse: TTTCCAAATCCTCGGCATAA	710

### Ethical consideration

The procedure was carried out based on the guidelines of the Ethics Committee of Urmia University, Faculty of Veterinary Medicine (Approval letter IRB protocol No: AECVU-185-2018).

### Statistical analysis

The variance normality and homogeneity of the data were evaluated by Kolmogorov-Smirnov and Levene's tests, respectively. Then, all the data were analyzed by one-way ANOVA with the appropriate post-hoc (Turkey's multiple comparisons).The appropriate analysis of covariance (ANCOVA) to analyze the relationship between cell number (as covariant) with mean alteration of genes expression. The SPSS software (Statistical Package for the Social Sciences, version 22.00, California, USA) was used for statistical and correlation analyses. A p < 0.05 was considered as a statistically significant and all data were presented as mean ± SD.

## 3. Results

### General findings 

Observations revealed no statistically significant difference in total body weight between all groups before and after the experiment. More analyses showed decreased testicular weight and size in PQ-sole group vs the control and other experimental groups (p < 0.02). Accordingly, the testicular weight relative to the total body weight was decreased in the PQ-sole group vs the control group. The animals in the PQ + CCN-treated group compared to the PQ-sole group represented more testicular weight to the total body weight ratio (Figures 1A, 1B, 1C, 1D, and 1E).

### Histological findings

Light microscopic analyses showed a remarkable (p < 0.01) increment in the percentage of seminiferous tubules with positive RI, TDI, and SPI in the PQ-sole group vs the control and other experimental groups. Meanwhile, the animals in the PQ + CCN-treated group exhibited ameliorated spermatogenesis (RI, TDI, and SPI) vs the PQ-sole group (p < 0.03, p < 0.01, and p < 0.02) (Figures 2B, 2C, and 2D). More histological analyses represented remarkable edema in the connective tissue of testicular tissue of the PQ-sole vs the control and other experimental groups (Figures 2A and 2E). Finally, the animals in the PQ + CCN-treated group exhibited increased numbers of Leydig and Sertoli cells *per* mm${}^{2}$ of tissue compared to the PQ-sole group (p < 0.02, p < 0.01) (Figures 2F and 2G).

### RT-PCR results

Semi quantitative RT-PCR showed that the mRNA levels of *bcl-2* and *caspase-3* decreased in the PQ + CCN-treated groups compared to the control and other experimental groups (p < 0.02 and p < 0.03). The mRNA level of *p53* was increased in the PQ-sole group vs the control and other experimental groups (p < 0.03) (Figures 3A, 3B, and 3C). To understand the subject, the total testicular cell numbers *per* mm${}^{2}$ of tissue in different groups and the correlation between the cellular number and mRNA levels were estimated. Observations represented a positive correlation between the mRNA levels and mRNA levels of *bcl-2*, *p53,* and *caspase-3* (Figures 3E, 3F, and 3G). Moreover, the covariance (ANCOVA) test was performed in which the cellular population of the tissue *per* mm${}^{2}$ act as the covariant. Observations showed a significant enhancement in the mRNA levels of *caspase-3*, and *p53* relative to cellular population (*per* mm${}^{2}$ of tissue) was decreased in the PQ + CCN-treated group vs the PQ-sole group. However, the mRNA level of *bcl-2* relative to cellular population (*per* mm${}^{2}$ of tissue) was increased in the PQ + CCN-treated group compared to the PQ-sole group (Figure 3H).

### Biochemical findings

The animals in CCN and PQ-sole groups exhibited diminished (p < 0.01) levels of SOD in comparison with the control and PQ + CCN-treated groups. Moreover, the animals in the PQ-sole group represented a remarkable (p < 0.01) increment in the testicular MDA content vs the control and other experimental groups (Figures 4A and 4B). In order to better understand the biochemical changes, the covariance (ANCOVA) test was performed in which the cellular population of tissue per mm${}^{2}$ act as the covariant. Observations showed a significant (p < 0.02) enhancement in tissue SOD level relative to testicular cellularity in the CCN-sole and PQ + CCN-treated groups vs the PQ-sole group (Figure 4C). The same results were obtained for the MDA contents of the testicles (Figure 4D).

### DNA ladder test

The PQ-induced DNA fragmentation was evaluated by DNA ladder test. The results showed that the PQ caused a violent DNA fragmentation. However, the animals in the CCN + PQ-treated group exhibited inhibited DNA fragmentation vs the PQ-sole group (Figure 5).

**Figure 1:** (A) Total body weight before and after the experiment; (B) Post and pre-experimental total body weight difference; (C) Photomicrograph of testes in the paraquat (PQ)-treated group vs the control group; (D) Post experiment testicular weight; and (E) Testicular weight relative total body weight. All data are presented as Mean ± SD.

**Figure 2:** (A) Photomicrograph of the testicular tissue; note intact spermatogenesis (I.SP) and spermiogenesis (I.S) in the control and crocin (CCN)-sole groups; GED: Germinal epithelium dissociation; AS: Arrested spermiogenesis; E: Edema; ASP: Arrested spermatogenesis. See ameliorated spermatogenesis (Am.S) and spermiogenesis in the PQ + CCN-treated group. H&E staining method, scale bar 120 µm. (B) Repopulation index (RI). (C) Tubular differentiation (TDI). (D) Spermiogenesis index (SPI). (E) Edema scores; +: Faint; ++: Moderate; and+++: Moderate-intensity; and ++++: intensive. (F) Leydig cell number *per* mm${}^{2}$ of tissue. (G) The Sertoli cell number *per* mm${}^{2}$ of tissue. All data are presented as Mean ± SD.

**Figure 3:** The RT-PCR electrophoresis and relative mRNA levels of (A) *bcl-2* to GAPDH, (B) *p53* to GAPDH, (C) *caspase-3* to GAPDH in different groups, and (D) the total cell number *per* mm${}^{2}$ in different groups. The correlations between (E) *caspase-3*, (F) *p53*, (G) *bcl-2,* and the total cell number *per* mm${}^{2}$. (H) Covariance (ANCOVA) test of mRNA levels of *caspase-3*, *bcl-2*, and *p53* relative to the total cell number per mm${}^{2}$ of tissue. All data are presented as Mean ± SD.

**Figure 4:** The testicular (A) Superoxide dismutase (SOD) and (B) Malondialdehyde (MDA) levels. The testicular (C) SOD and (D) MDA levels relative to total cell number per mm${}^{2}$. All data are presented as Mean ± SD.

**Figure 5:** DNA laddering test; the lane paraquat (PQ)-treated group represents severe DNA fragmentation, which is ameliorated in crocin (CCN)-treated groups (G4 and G5).

## 4. Discussion

Our findings showed that the PQ significantly downregulated the spermatogenesis indices, suppressed testicular SOD status, increased lipid peroxidation ratio, enhanced *p53* and *capsapse-3* expression, downregulated *bcl-2* expression, and resulted in severe DNA damage. However, the CCN ameliorated the PQ-induced impairments, including spermatogenesis, spermiogenesis, testicular SOD level, and MDA content, *bcl-2*, *p53*, and *caspase-3* expressions and significantly inhibited the PQ-induced DNA fragmentation. The oxidative stress, caused by pathologically produced ROS, is considered as one of the main reasons for spermatogenesis arrest (5). A study showed that the oxidative stress (OS) causes to damage the reproductive system and sperm quality, therefore followed by reducing sperm motility, lipid peroxidation, and increasing the sperm DNA damage (31). Some other studies also showed that ROS had considerable effects on spermatogenesis and sperm function and apoptosis (32, 33). A study showed that oxidative stress induced by TD in adult rats caused the Johnson's score, mean seminiferous tubule diameter (MSTD) and height (thickness) of seminiferous tubule epithelium (HSTE) were significantly ameliorated with the administration extract of *Fumaria parviflora* (FP). The gene expression of *bcl-2*, the level of serum testosterone hormone and antioxidant parameters —GPx and SOD— also were significantly higher in the FP-receiving groups than TD group (34). These results are accommodated to present study that showed all destructive effects of oxidative stress induced by PQ were significantly ameliorated by the administration of CCN. Another study also revealed that the administration of an antioxidant such as onion juice could enhance the quality of sperm and fertility power after testicular TD (35). Then, the previous investigations confirm the results of the present study in the beneficial effects of antioxidants as a major therapeutic role against the oxidative stress-inducing agents. Accordingly, the imbalanced and/or pathologically produced ROS are capable to negatively affect the DNA, RNA, lipid, and protein contents of germinal and somatic cells in testicular tissue and by administrating different antioxidants, it is possible to fairly ameliorate the ROS-induced damage (36). In line with this issue, our findings showed a significant enhancement in MDA and decreased SOD contents as well as diminished RI, DI, and SPI indices in the PQ-sole group. However, the CCN-treated group (PQ + CCN-treated) exhibited ameliorated antioxidant status and spermatogenesis indices. Thus, as a preliminary outcome, the PQ by downregulating the testicular antioxidant capacity depressed the spermatogenesis process (Figures 4C and 4D). However, in order to understand how exactly the CCN maintained spermatogenesis, one should note that the mitochondria are the main sources and/or victims of ROS. In fact, the respiratory chain of mitochondria powerfully produces ROS, which potentially is able to promote excessive ROS generation ending with oxidative stress and/or mitochondrial membrane disintegration, especially when the antioxidant status is suppressed (37). On the other hand, it should be considered that different types of mitochondrial SODs play an essential role in neutralizing the respiratory chain-derived ROS by catalyzing the superoxide anion dismutation via oxidation-reduction of the transition metal at the enzyme's active site (38). In this line, the MnSOD converts the superoxide to hydrogen peroxide, which is consequently metabolized by glutathione peroxidase (Gpx1). Moreover, smaller cell types contain CuZnOD in the mitochondrial intermembrane space, which converts the O${}_{2}^{-}$ to H${}_{2}$O (39). In addition, previous findings have shown the antioxidant properties of CCN. Accordingly, Bakhtiary and co-workers have reported that the CCN fairly downregulates the oxidative stress, upregulates the sperm quality, and consequently improves the in-vitro fertilization ratio in cyclophosphamide-induced animals (26). Another study by Dar and co-workers has shown that the antioxidant property and lipid peroxidation inhibition capacity of CCN are related to the hydroxyl and glucose moieties, which are known as necessary radical scavenger components (40).

Turning back to the relation between oxidative stress and mitochondria-dependent apoptosis, one should consider that the ROS-induced lipid peroxidation adversely affects the mitochondrial metabolism, vital functions, including respiration and oxidative phosphorylation, inner membrane barrier properties, and maintenance of mitochondrial membrane potential (41). In line with this issue, the *bcl-2*, as stabilizing the protein in the mitochondrial membrane, is involved in maintaining the membrane integrity. Thus, any reduction in *bcl-2* expression and/or the interaction of lipid peroxidation products with *bcl-2* trigger the mitochondrial membrane disintegration (42). Accordingly, the *bcl-2* and *bcl-xL* in the mitochondria prevent the apoptogenic factors, including cytochrome c and/or apoptosis-inducing factor (AIF) release from mitochondrial inter-membrane space into the cytoplasm because the released cytochrome c and AIF directly activate the caspases, as finishers of the apoptosis pathway (43). Our findings showed that the CCN significantly upregulated the *bcl-2* expression and remarkably diminished the *caspase-3* expression in the PQ + CCN-treated group. On the other hand, the animals in the PQ + CCN-treated group exhibited diminished DNA damage (hall mark of apoptosis) as well. Taking together, we can come close to this fact that upregulation of antioxidant potential simultaneous with enhanced expression of *bcl-2* in the CCN-treated group inhibited the intrinsic apoptosis pathway by maintaining the mitochondrial membrane integrity.

Aside from all possible mechanisms and/or pathways discussed earlier, the *p53*-dependent checkpoint activity stops cell cycle in mitotically dividing germ cells with DNA double-strand breaks (DSBs). Indeed, the DSBs trigger the *p53* expression, which in turn initiates the DNA repairing pathways. When the DNA damage is present before entry into S phase, *p53* halts the cell cycle in G1 stage via *p21* (cyclin-dependent kinase inhibitor *cdkn1a*)-dependent pathway (44). However, considering the decreased DNA fragmentation and diminished expression of *p53* in the PQ + CCN-treated group, we can suggest that CCN could fairly diminish the DNA damage and as a consequent could potentially inhibit DNA damage. The limitations of our work suggests future studies in this field to investigate on the probability of the direct role of PQ on testis and evaluating the ultrastructure of the blood testes barrier in PQ poisoning. Moreover, the probable effects of PQ and CCN on hypothalamus-hypophyses and gonadal axis in molecular and gene expression level.

## 5. Conclusion

This study showed that the antioxidant properties of CCN can be able to protect the testes against the oxidative stress induced by PQ histologically and histomorphometrically. Furthermore, the CCN by upregulating the SOD activity diminishes the lipid peroxidation ratio and by enhancing the *bcl-2* expression maintains the mitochondrial membrane integrity. This trend results the maintaining of DNA integrity by CCN and inhibits the *p53* and *caspase-3* expressions. All these findings suggest that, in addition to CCN-induced antioxidant property, it has the ability to fairly inhibit the PQ-induced intrinsic apoptosis as well.

##  Conflict of Interest

The authors have no conflicts of interest to declare.
